# Deep-Learning-Based Survival Prediction of Patients in Coronary Care Units

**DOI:** 10.1155/2021/5745304

**Published:** 2021-12-24

**Authors:** Rui Yang, Tao Huang, Zichen Wang, Wei Huang, Aozi Feng, Li Li, Jun Lyu

**Affiliations:** ^1^Clinical Research Center, The First Affiliated Hospital of Xi'an Jiaotong University, Xi'an, Shaanxi 710061, China; ^2^School of Public Health, Xi'an Jiaotong University Health Science Center, Xi'an, Shaanxi 710061, China; ^3^Department of Clinical Research, The First Affiliated Hospital of Jinan University, Guangzhou, Guangdong 510630, China; ^4^Department of Public Health, University of California, Irvine, CA 92697, USA; ^5^Department of Hepatobiliary Surgery II, Meizhou People's Hospital, Meizhou, Guangdong 514031, China

## Abstract

**Background:**

A survival prediction model based on deep learning has higher accuracy than the CPH model in predicting the survival of CCU patients, and it also has a better discrimination ability. We collected information on patients with various diseases in coronary care units (CCUs) from the Medical Information Mart for Intensive Care III (MIMIC-III) database. The purpose of this study was to use this information to construct a neural-network model based on deep learning to predict the survival probabilities of patients with conditions that are common in CCUs.

**Method:**

We collected information on patients in the United States with five common diseases in CCUs from 2001 to 2012. We randomly divided the patients into a training cohort and a testing cohort at a ratio of 7 : 3 and applied a survival prediction method based on deep learning to predict their survival probability. We compared our model with the Cox proportional-hazards regression (CPH) model and used the concordance indexes (C-indexes), receiver operating characteristic (ROC) curve, and calibration plots to evaluate the predictive performance of the model.

**Results:**

The 3,388 CCU patients included in the study were randomly divided into 2,371 in the training cohort and 1,017 in the testing cohort. The stepwise regression results showed that the important factors affecting patient survival were the type of disease, age, race, anion gap, glucose, neutrophils, white blood cells, potassium, creatine kinase, and blood urea nitrogen (*P* < 0.05). We used the training cohort to construct a deep-learning model, for which the C-index was 0.833, or about 5% higher than that for the CPH model (0.786). The C-index of the deep-learning model for the test cohort was 0.822, which was also higher than that for the CPH model (0.782). The areas under the ROC curve for the 28-day, 90-day, and 1-year survival probabilities were 0.875, 0.865, and 0.874, respectively, in the deep-learning model, respectively, and 0.830, 0.843, and 0.806 in the CPH model. These values indicate that the survival analysis model based on deep learning is better than the traditional CPH model in predicting the survival of CCU patients.

**Conclusion:**

A survival prediction model based on deep learning has higher accuracy than the CPH model in predicting the survival of CCU patients, and it also has a better discrimination ability.

## 1. Introduction

Cardiovascular diseases, which include acute myocardial infarction (AMI), arrhythmia, and other cardiovascular diseases, have always been important life-threatening conditions for patients. These diseases have the characteristics of high prevalence, high disability, and high mortality. The number of deaths due to cardiovascular disease in the world reaches 15 million every year, ranking first among various causes of death. The treatment and prognosis of cardiovascular diseases have always been the focus of research.

In the late 1960s, the coronary care units (CCUs) were established specifically for the research and treatment of cardiovascular disease [1–3]. CCUs have been widely implemented since Killip and Kimball first reported that the use of a CCU could reduce mortality by nearly 20% [4]. After a long period of development, the survival rate in CCUs has increased from 18–20% to 40–46% over several decades, demonstrating the effectiveness of these units [5–7]. Studying the main factors that affect the survival of CCU patients provides modern CCUs with more mortality information, which helps to determine the main factors that affect the survival of patients, thereby improving the standard of care for patients in these units [3].

As a statistical method, survival models are commonly used in clinical research to identify potential risk factors and predict the risk of various clinical outcomes, including the overall survival of patients with various diseases (e.g., cancer). The Cox proportional-hazards regression (CPH) model [8] is one of the most commonly used survival analysis tools [9, 10]. It is a semiparametric model that can be used to calculate the impact of characteristics (independent variables) on the risk of specific events (e.g., death), such as the effect of tumor size on the risk of death [11–13]. CPH-based survival models can help clinicians make more-personalized treatment decisions for individual patients. The traditional CPH model assumes that each independent variable has a linear effect on the model over time [14, 15]. However, in many cases, this linearity assumption will oversimplify the relationship between predictors and prognosis, especially in cancer diseases with a poor prognosis [16]. At the same time, data with high nonlinearity, high dimensionality, and from small samples will bring computational challenges. Deep-learning-based methods integrate clinical data into neural networks and provide powerful nonlinear capabilities to survival forecasts [17]. Deep learning will provide more complex and accurate algorithm support for survival analysis and may result in more practical predictive models.

This study was based on a large amount of medical data from the intensive disease database (MIMIC-III database), which aimed to develop a deep learning model to predict the mortality of CCU patients and to provide a theoretical basis and model basis for their treatment and prognosis.

## 2. Methodology

Figure 1 outlines the general flow of this research, whose main steps were data extraction, data preprocessing, model training, and model evaluation. Specifically, the Multiparameter Intelligent Monitoring in Intensive Care III (MIMIC-III) database [18] was investigated. PostgreSQL [19] and SQL [20] were used for data extraction, the Acute Physiological Score III (APS-III) and Sequential Organ Failure Assessment (SOFA) score were calculated, and Python [21] was used for data preprocessing [22] and model evaluation. We used the PyTorch deep-learning framework [23] to construct the neural network, and Python and R [24] were used for data visualization. The experiments were run on an NVIDIA GTX1050 GPU.

### 2.1. Data Extraction

All patient data included in this study were obtained from the MIMIC-III database [18]. This is a large public database that contains anonymous health-related information related to more than 40,000 patients who stayed in the intensive care units (ICUs) of Beth Israel Deacon Medical Center between 2001 and 2012 [18, 25]. The database includes demographic information, vital-sign measurements made at the bedside (approximately one data point per hour), laboratory test results, procedures, medications, caregiver care, imaging reports, and mortality information (in-hospital and during hospitalization). Through the registration website, we obtained the relevant certificate and applied for and signed the agreement to obtain the right to use the data. Referring to the official tutorial for establishing a PostgreSQL database, SQL was used to identify all CCU patients in the database and obtain relevant data.

### 2.2. Data Preprocessing

We extracted the relevant data on CCU patients, including their physiological index data, as detected by the CareVue and MetaVision systems from the constructed MIMIC-III database. The data table stores the original values recorded by medical staff or obtained during system monitoring, which need to be summarized and processed before they can be applied to the model. We first summarized the patient indicators of two monitoring systems, counted the number of patients with different diseases, and selected the five most-representative diseases with the largest number of patients for inclusion in this research. The patient's survival time and survival status were included in the prediction method.

### 2.3. Research Method

The patient data extracted from the MIMIC-III database were grouped according to the disease, and the five disease states with the largest number of patients and relevant health records were selected for the analyses. The five disease states were AMI, heart failure, tachycardia, respiratory failure, and valve disorder. Related health records were also obtained, including age, sex, race, heart rate, respiratory rate, body temperature, systolic blood pressure, diastolic blood pressure, oxygen saturation, neutrophils, lymphocytes, white blood cells, platelets, hemoglobin, anion gap, bicarbonate, chloride, glucose, sodium, potassium, hematocrit, creatine kinase, and blood urea nitrogen.

We grouped the data indicators according to their standard physiological standard ranges and then used the CPH model and stepwise regression analysis to determine the baseline clinical characteristics related to survival status, which revealed nine characteristics with statistically significant hazard ratios (HRs). Considering clinical factors, we finally chose age, race, anion gap, glucose, neutrophils, white blood cells, potassium, creatine kinase, and blood urea nitrogen as predictors. The SOFA score and simplified APS-III were calculated according to the official codes in the MIMIC-III database, and they were incorporated into the model as variables. The patient survival time was calculated based on the date of death from the social security database (dod_ssn from table PATIENTS.csv) and the admission time (ADMITTIME from table ADMISSIONS.csv) and with a survival indicator of 1. If there was no time to death, the longest recorded time of monitoring care was taken as the patient's survival time (90 days or 4 years), with a survival indicator of 0.

We then used the selected features to construct a survival analysis model, comprising a deep-learning neural-network model with three hidden layers. We compared the deep-learning model with the CPH model, calculated their C-indexes and areas under the receiver operating characteristic (ROC) curves (AUCs) in the testing cohort to evaluate their judgment and discrimination abilities, and drew a calibration plot to evaluate the consistency of the model.

### 2.4. Statistical Analysis

We first performed a descriptive statistical analysis of the data of CCU patients. Continuous variables were expressed as the median (25th to 75th percentile) values (because they were not normally distributed), and categorical variables were expressed as percentages. The patients were randomly assigned to the training cohort (70%) or testing cohort (30%) for model construction and validation. The backward stepwise selection method was then applied to the CPH model with the training cohort to select variables. The accuracy of the model was evaluated using the C-index and AUC. A calibration plot was used to evaluate the agreement between the labeling results and the predicted probabilities.

### 2.5. Model Design

Our model is based on the mainstream deep-learning framework PyTorch, comprising a feed-forward neural network with three hidden layers (Figure 2). We used to represent the clinical feature predictor variable, with *m* = 16, *k* = 16, and *l* = 8, and we finally output the patient's risk value. Batch normalization, a nonlinear activation layer, and a dropout layer were used between each hidden layer in order to increase the fitting ability of the model.

## 3. Results

### 3.1. Patient Characteristics

Table 1 lists the baseline characteristics of patients in the training and testing cohorts. The training cohort included 2,371 patients admitted to the CCUs unit, comprising 1,479 males (62.4%) and 892 females (37.6%) with a mean age of 70 years.

The first diagnosis of these patients was predominantly MI (*n* = 1,477, 62.3%), followed by heart failure (*n* = 498, 21%), tachycardia (*n* = 164, 6.9%), respiratory failure (*n* = 132, 5.2%), and valve disorder (*n* = 109, 4.6%). A log-rank test used to assess differences between the two cohorts produced *P* = 0.730, indicating no significant difference in the survival curves between the two cohorts and a balanced data distribution. The Kaplan-Meier analysis curve of the train and test cohorts is shown in Figure 3.

### 3.2. Variable Screening

The age at diagnosis, current age, sex, race, anion gap, glucose, neutrophils, white blood cells, potassium, creatine kinase, blood urea nitrogen, APS-III, and SOFA score were entered into the multivariate CPH analysis.  Table 2 lists the results of the multivariate CPH analysis. Combining the basic data statistics in Table 1 and multivariate CPH survival analysis showed that CCU mortality was not correlated with patient sex, whereas patients with heart failure (HR = 1.508, *P* < 0.001), tachycardia (HR = 1.598, *P* = 0.001), and respiratory failure (HR = 1.984, *P* < 0.001) had higher risks of death compared with MI patients. Compared with white race, patients classified as Hispanic (HR = 1.647, *P* = 0.080) and unknown race (HR = 1.446, *P* < 0.001) had higher risks of death. The following indicators were positively correlated with a higher risk of death: anion gap (<18 and >16 mmol/L), glucose (>140 g/dL), white blood cells (>10 × 10^9^/L), potassium (<3.5 and >5.5 mmol/L), creatine kinase (<18 and >198 U/L), and blood urea nitrogen (>22 mg/dL). Age, APS-III, and SOFA score were also positively correlated with the risk of death.

### 3.3. Cox Proportional-Hazards Regression Model and Deep-Learning Model in the Training and Testing Cohorts

The performance of survival prediction based on deep learning was compared with the CPH model using the testing cohort. The performance of these two models was compared using Harrell's C-index, which measures the consistency between the predicted risk and actual survival. The training and testing results for the deep-learning model are shown in Figure 4. We stopped training in advance to avoid overfitting and obtain the best model. The deep-learning survival model performed best, with C-indexes in the training and testing cohorts of 0.833 and 0.822, respectively, while they were 0.786 and 0.782 for the CPH model.

### 3.4. Comparison between the Deep-Learning Model and the Cox Proportional-Hazards Regression Model

The calibration plot in Figure 5 shows that compared with the CPH model, the 28-day, 90-day, and 1-year probability standard curves of the deep-learning model were very close to the standard 45-degree diagonal, which indicates that the new model is well calibrated.

We calculated the 28-day, 90-day, and 1-year ROC curves of the two models to verify their discrimination abilities.  Figure 6 shows the overall performance of the survival analysis model. The AUCs for the 28-day, 90-day, and 1-year survival probabilities were 0.875, 0.865, and 0.874, respectively, for the deep-learning model, and 0.830, 0.843, and 0.806 for the CPH model. It indicates that the deep learning model is more accurate and has better classification discrimination in predicting the survival prognosis of CCU patients.

## 4. Discussion

In this study, we developed and verified an accurate deep learning model for predicting the risk of death in CCU patients. Because the traditional regression model predicts mortality rate based on a simplified relationship between predictor variables and prognosis, it is difficult to improve the predictive ability of that model. Therefore, based on the strong nonlinear fitting ability and more precise algorithms of deep learning, we constructed a neural-network model for predicting the survival rate of patients in the CCUs and explored the influencing patient factors.

Previous studies found that the in-hospital mortality rates of CCU patients were in the range of 5.6–15.2% [3, 26]. Although developments in modern medical technologies have significantly decreased the mortality rate of CCU patients, the survivors in CCUs still have a high disability rate. Analyzing the survival of CCU patients and understanding the influencing factors will help clinicians to choose treatment options, improve survival rates, and avoid unnecessary treatments [10, 11]. Considering that the CPH model is currently one of the most widely used models for predicting the prognosis of various diseases, but the CPH model has some inherent algorithmic flaws. In this study, a more complex and accurate deep learning model was selected for comparison with the CPH model. It is to build a model that is more suitable for predicting the mortality of CCU patients.

Under the guidance of clinicians and previous studies, we have included variables related to mortality in CCU patients, which are easily available clinically to improve the usability of the model. After further analysis and variable selection, the experimental results show that the neural-network model based on deep learning showed better prediction performance than the traditional semiparametric CPH model. The C-index showed that the accuracy of the deep-learning model (0.822) was about 4% better than that of the CPH model (0.782). It was indicated that deep learning may be more suitable for handling large samples, multivariate and nonlinear survival analysis than the CPH model, which was consistent with the research results [27–29].

The severe lack of data on critically ill patients is already well known. In order to better study the treatment and prognosis of CCU patients, we chose to use the MIMIC database, which is difficult but with a large amount of data on critically ill patients, as the data source for the study, which ensures the reliability of the entire study results. All the C-indexes shown in the results are close to 1, which shows that the model constructed in this study has good judgment ability and is better than the model reported in the related literature [30–32]. The result of the calibration curve shows that this study still has a high consistency.

It can be seen from the risk factors (i.e., age, race, anion gap, glucose, neutrophils, white blood cells, potassium, creatine kinase, blood urea nitrogen, APS-III, and SOFA score) that are finally incorporated into the predictive model. Although the current clinical scores have the greatest impact on the prediction results, it is not the most suitable score for patients with CCUs. Our model is improved on the basis of the existing clinical scores and is more suitable for the prognosis prediction of CCU patients. At the same time, some recognized risk factors that affect the outcome of CCU patients, such as age, glucose, and creatine kinase, are also included in the model constructed in this study, which also reflects the reliability of the model. Of course, all the risk factors in the model have strong clinical accessibility, which also provides convenience for patients and medical staff to use.

This research was subject to some limitations. First, it only included CCU patients from a single center, and hence, the obtained results might not be generalizable to other populations. Utilizing larger datasets from multiple centers may provide more-reliable results and further establish the effectiveness of deep-learning-based survival prediction in CCU patients. Second, we only selected more-serious diseases in the CCUs, and so the overall predictions may be biased, reducing the prognostic ability of the new model in some patients with rare diseases. It is necessary to find a better way to establish a unified model for different diseases to predict the overall survival of CCU patients. Finally, due to the inexplicability of deep-learning models, the prediction process is a black-box model, which is not conducive to understanding the impact of each included factor. An interpretable neural-network model and higher accuracy AUC score are a feasible research direction in the future.

## 5. Conclusion

This study first used stepwise regression analysis to determine the risk factors that affect the prognosis of CCU patients and then constructed a three-layer neural network prediction model based on these risk factors. The findings demonstrate that the deep-learning model can provide good predictions for the prognosis of CCU patients, with its performance ability being better than that of the CPH prediction model.

## Figures and Tables

**Figure 1:** Work flow overview.

**Figure 2:** Neural network model structure diagram.

**Figure 3:** Kaplan-Meier curve of training and testing sets. There was no statistically significant difference between the survival of training and testing sets in the log-rank test (*P* = 0.73).

**Figure 4:** The loss and C-index change process diagram of training and testing.

**Figure 5:** Calibration plot. Calibration plot of the (a) CPH model and (b) deep learning model for 28-day, 90-day, and 1-year prediction in testing cohort population.

**Figure 6:** ROC plot. Comparison of ROC between the CPH model and the deep learning model in (a) 28 days, (b) 90 days, and (c) 1 year in testing cohort population.

**Table 1:** Baseline demographic and laboratory characteristics of patients.

Variable	Training cohort	Testing cohort	*P*
	(*n* = 2371)	(*n* = 1017)	
*Disease (%)*			0.742
Myocardial infarction	1477 (62.3)	629 (61.8)	
Heart failure	498 (21.0)	226 (22.2)	
Tachycardia	164 (6.9)	67 (6.6)	
Respiratory failure	123 (5.2)	44 (4.3)	
Valve disorder	109 (4.6)	51 (5.0)	
*Race (%)*			0.321
White	1659 (70.0)	698 (68.6)	
Black	136 (5.7)	64 (6.3)	
Asia	27 (1.1)	13 (1.3)	
Hispanic	34 (1.4)	25 (2.5)	
Others	50 (2.1)	26 (2.6)	
Unknown	465 (19.6)	191 (18.8)	
*Anion gap (mEq/L, %)*			0.104
8~16	1092 (46.1)	464 (45.6)	
<8	130 (5.5)	39 (3.8)	
>16	1149 (48.5)	514 (50.5)	
*Glucose (mg/dL, %)*			0.377
70~140	1481 (62.5)	658 (64.7)	
<70	45 (1.9)	15 (1.5)	
>140	845 (35.6)	344 (33.8)	
*Neutrophil (%)*			0.868
50~70	366 (15.4)	163 (16.0)	
<50	50 (2.1)	23 (2.3)	
>70	1955 (82.5)	831 (81.7)	
*White blood cell (K/uL, %)*			0.611
4~10	1947 (82.1)	838 (82.4)	
<4	5 (0.2)	4 (0.4)	
>10	419 (17.7)	175 (17.2)	
*Potassium (mEq/L, %)*			0.659
3.5~5.5	1933 (81.5)	841 (82.7)	
<3.5	4 (0.2)	1 (0.1)	
>5.5	434 (18.3)	175 (17.2)	
*Creatine kinase (%)*			0.013
18~198	1126 (47.5)	529 (52.0)	
<18	17 (0.7)	2 (0.2)	
>198	1228 (51.8)	486 (47.8)	
*Blood urea nitrogen (mg/dL, %)*			0.869
6~22	764 (32.2)	320 (31.5)	
<6	11 (0.5)	4 (0.4)	
>22	1596 (67.3)	693 (68.1)	
*Sex* = *male*/*female(%)*	1479/892 (62.4/37.6)	609/408 (59.9/40.1)	0.183
*Age (median [IQR])*	70 [59,79]	70 [59,79]	0.769
*APS-III score (mean (SD))*	42.80 (19.38)	42.12 (18.94)	0.348
*SOFA score (mean (SD))*	3.76 (2.93)	3.76 (2.96)	0.976
*Status* = *alive*/*dead(%)*	1311/1060 (55.3/44.7)	568/449 (55.9/44.1)	0.794

**Table 2:** Selected variables by multivariable Cox regression analysis.

Multivariate analysis			
Variables	HR	95% CI	*P* value
*Disease*			
Myocardial infarction	Reference		
Heart failure	1.508	1.275-1.785	<0.001
Tachycardia	1.598	1.213-2.106	0.001
Respiratory failure	1.984	1.557-2.528	<0.001
Valve disorder	0.947	0.66-1.359	0.768
*Race*			
White	Reference		
Black	0.988	0.745-1.309	0.931
Asia	0.752	0.399-1.419	0.379
Hispanic	1.647	0.942-2.880	0.080
Others	0.531	0.314-0.897	0.018
Unknown	1.446	1.241-1.686	<0.001
*Sex*			
Male	Reference		
Female	1.019	0.897-1.156	0.777
*Anion gap (mmol/L)*			
8~16	Reference		
<8	1.356	1.018-1.807	0.038
>16	1.253	1.090-1.439	0.001
*Glucose (g/dL)*			
70~140	Reference		
<70	0.86	0.574-1.289	0.466
>140	1.173	1.031-1.333	0.015
*White blood cell (X109/L)*			
4~10	Reference		
<4	1.459	0.358-5.945	0.598
>10	1.454	1.246-1.696	<0.001
*Neutrophil (%)*			
50~70	Reference		
<50	0.639	0.395-1.034	0.068
>70	0.852	0.704-1.032	0.101
*Potassium (mmol/L)*			
3.5~5.5	Reference		
<3.5	22.994	7.262-72.808	<0.001
>5.5	1.215	1.048-1.410	0.01
*Creatine kinase (U/L)*			
18~198	Reference		
<18	2.255	1.246-4.079	0.007
>198	0.856	0.744-0.984	0.029
*Blood urea nitrogen (mg/dL)*			
6~22	Reference		
<6	1.066	0.393-2.892	0.899
>22	1.584	1.312-1.913	<0.001
*Age*	1.030	1.024-1.036	<0.001
*APS-III*	1.021	1.016-1.026	<0.001
*SOFA*	1.054	1.022-1.088	0.001

## Data Availability

The datasets used and/or analyzed during the current study are available from the MIMIC-III official (https://mimic.mit.edu/).

## Abbreviations

CCUs: Coronary care units
MIMIC-III: Medical Information Mart for Intensive Care III
CPH: Cox proportional-hazards regression
C-index: Concordance indexes
ROC: Receiver operating characteristic
AMI: Acute myocardial infarction
APS-III: Acute Physiological Score III
SOFA: Sequential Organ Failure Assessment
ICUs: Intensive care units
ROC: Receiver operating characteristic.
